The article "Effect of miR-488 on Colon Cancer Biology and Clinical Applications" was retracted in 2023. Reasons: signs of a paper mill; compromised peer review; unreliable results or conclusions.

# Effect of miR-488 on Colon Cancer Biology and Clinical Applications

**DOI:** 10.1155/2022/2138954

**Published:** 2022-05-05

**Authors:** Liangqin Wu, Songguo Li, Peng Shu, Qian Liu

**Affiliations:** ^1^Department of Gastroenterology, Anhui No.2 Provincial People's Hospital, Hefei, Anhui, China; ^2^Department of Pathology, Anhui No.2 Provincial People's Hospital, Hefei, Anhui, China; ^3^Department of Pathology, The Affiliated Suzhou Hospital of Nanjing Medical University, Suzhou Municipal Hospital, Nanjing, Jiangsu, China

## Abstract

**Objective:**

To explore the expression levels of miR-488, miR-29c-3p, and growth differentiation factor 15 (GDF15) in colon cancer tissue and analyze their relationship with clinicopathological features in patients with colon cancer.

**Methods:**

The study was conducted from November 2012 to November 2020. A total of 200 patients with colon cancer were treated in our hospital during this period. During the operation, the colon cancer tissues and the adjacent tissues whose distance from the cancer tissues were more than 5 cm were collected, and the expression levels of miR-488, miR-29c-3p, and GDF15 mRNA in colon cancer tissues were detected by qRT-PCR (real-time fluorescence quantitative). The relationship between them and the clinicopathological features and prognosis of patients with colon cancer were analyzed and discussed.

**Results:**

The level of miR-488 in colon cancer tissues was lower than that in adjacent tissues, but the levels of miR-29c-3p and GDF15 mRNA in colon cancer tissues were higher than those in adjacent tissues (*P* < 0.05). Compared with paracancerous tissues, the expression rates of miR-29c-3p and GDF15 protein were higher in colon cancer tissues (*P* < 0.05). There was no difference in age, sex, tumor location, and tumor diameter between high expression of miR-488 group and low expression of miR-488 group (*P* > 0.05). The degree of differentiation, depth of invasion, TNM stage, lymph node metastasis, and other factors have a direct impact on the level of miR-488 and the expression of miR-29c-3p (*P* < 0.05). The depth of invasion, TNM stage, and lymph node metastasis could affect the expression of GDF15 in patients with colon cancer (*P* < 0.05).

**Conclusion:**

miR-488, miR-29c-3p, and GDF15 in colon cancer tissue are related to the clinicopathological features of patients in varying degrees and may become markers after early warning of colon cancer, which can provide effective guidance for clinical diagnosis and treatment.

## 1. Introduction

Colon cancer is a common digestive tract malignant tumor that occurs in the colon, which usually occurs at the junction of rectum and sigmoid colon [1, 2]. The incidence of colon cancer is the highest in the age group of 40 to 50 years old, the ratio of men and women is 2∼3: 1 [3]. The incidence rate occupies the third place of gastrointestinal tumors [4, 5]. Colon cancer is mainly adenocarcinoma, mucinous adenocarcinoma, and undifferentiated carcinoma [6]. The general shape is polyp, ulcer, etc. [7]. Colon cancer can develop around the intestinal wall, spread up and down the longitudinal diameter of the intestinal canal, or infiltrate deeply into the intestinal wall. In addition to lymphatic vessels, blood flow metastasis, and local invasion, colon cancer can also be implanted into the abdominal cavity or spread and metastasize along sutures and incisions [8]. Patients with chronic colitis, patients with colonic polyps, and obese men are susceptible people. Moreover, related research shows that the number of men in colon cancer patients is higher than that of women [9–11]. Although people have conducted more in-depth research on the diagnosis and treatment of colon cancer, the number of patients with colon cancer is still increasing due to changes in people's lifestyle and diet [12, 13]. Therefore, it is of positive significance to explore the relevant factors in the development of colon cancer disease so as to effectively prevent the disease [14, 15]. According to related studies, the expression of miR-488 is low in non-small cell lung cancer cells, and if it is overexpressed, it can reduce the proliferation and renewal ability of cancer cells [16, 17]. miR-29c-3p is a potential marker of poor prognosis, and its high expression in human hepatocellular carcinoma is closely related to high clinical stage and low survival rate [18]. The positive expression rate of GDF15 (growth differentiation factor 15) in gastric cancer was significantly higher than that in normal gastric mucosa, which was closely related to the degree of differentiation and lymph node metastasis of gastric cancer [19]. A study reports that aging-related tissue microenvironment promotes the formation of colon cancer by secreting factor GDF15 [11]. This paper analyzes the expression of the abovementioned indexes in the tissues of patients with colon cancer, hoping to provide some guidance for related research in the future.

The article "Effect of miR-488 on Colon Cancer Biology and Clinical Applications" was retracted in 2023. Reasons: signs of a paper mill; compromised peer review; unreliable results or conclusions.

## 2. Materials and Methods

### 2.1. General Information

This study has been approved by the Ethics Committee of Anhui No.2 provincial people's hospital, and the retrospective study time is from November 2012 to November 2020, and 200 patients with colon cancer treated in our hospital during this period were taken as the main observation objects of this study. All the 200 patients in the group understood the content of this study and participated voluntarily. Among them, there were 114 males and 86 females, aged from 35 to 72 years old, with an average age of (54.28 ± 6.37) years.

Inclusion criteria are as follows: (1) after pathological examination, the patient was diagnosed as primary colon cancer, (2) before entering the group, the patients had not received chemotherapy, radiotherapy or operation, (3) the clinical data of the patients were complete, and (4) the patient signed an informed consent form with his or her family.

Exclusion criteria are as follows: (1) the patients had serious deficiency of heart, liver, kidney, and other functions; (2) the patients were complicated with tumors in other locations; and (3) the patient has mental system disease or is unable to communicate effectively because of language barrier.

### 2.2. Research Methods

The medical staff should collect the colon cancer tissue and the paracancerous tissue during the operation of the patients and pay attention to the distance between the paracancerous tissue and the cancer tissue above 5 cm. Some of them were frozen in liquid nitrogen and stored in refrigerator at −80°C for qRT-PCR test. The other part was first soaked in formaldehyde (4%) and then made into paraffin sections with a thickness of 4 *μ*m, which were used for immunohistochemical staining.

After discharge, patients need to be followed up by telephone or re-examination, ask about their survival, and record in detail.

### 2.3. Observation Index

The relative expression of miR-488, miR-29c-3p, and GDF15 mRNA in different colonic tissues was detected by qRT-PCR. Expression of GDF15 protein in different colonic tissues was measured by enzyme-linked immunosorbent assay (ELISA).

### 2.4. Statistical Analysis

Reporting the data analysis section, the statistical software SPSS24.0 was used to process, count data are indicated as ($\bar{x}\pm s$), the test is performed by *t*-test, the counting data are expressed by *n* (%), and the chi-square test is used for inspection. If there is a *P* < 0.05, it shows that there is a significant difference between the two groups.

## 3. Result

### 3.1. Relative expression of miR-488, miR-29c-3p, and GDF15 mRNA in different colonic tissues

The levels of miR-488, miR-29c-3p, and GDF15 mRNA in colon cancer tissues were compared with those in adjacent tissues. It was found that the levels of miR-488 in colon cancer tissues were lower than those in adjacent tissues, but the levels of miR-29c-3p and GDF15 mRNA in colon cancer tissues were higher than those in adjacent tissues. There was significant difference between groups, *P* < 0.05. Details are shown in Table 1.

### 3.2. Expression of miR-29c-3p and GDF15 in different colonic tissues

The expression of miR-29c-3p mainly existed in cells, and the expression rate in colon cancer tissues was higher than that in paracancerous tissues, and there was significant difference between the two groups (*P* < 0.05). The expression of GDF15 protein was significantly higher in the cytoplasm and nucleus, and also higher in the colon cancer tissues than in the paracancerous tissues (*P* < 0.05). Details are shown in Table 2.

The article "Effect of miR-488 on Colon Cancer Biology and Clinical Applications" was retracted in 2023. Reasons: signs of a paper mill; compromised peer review; unreliable results or conclusions.

### 3.3. Relationship between miR-488, miR-29c-3p, and GDF15 protein levels and clinicopathological features of colon cancer

The average expression level of miR-488 was 0.69. According to this standard, the patients could be divided into two groups: high expression of miR-488 (*n* = 118) and low expression of miR-488 (*n* = 82). The related factors that may affect the level of miR-488, miR-29c-3p, and GDF15 protein in colon cancer tissues were compared. It was found that age, sex, tumor location, tumor diameter, and other factors had no effect on the related indexes of colon cancer, and there was no difference between the two groups (*P* > 0.05), as detailed in Table 3. According to the expression levels of miR-29c-3p, the patients could be divided into two groups: high expression (*n* = 113) and low expression (*n* = 87). The degree of differentiation, depth of invasion, TNM stage, lymph node metastasis, and other factors have a direct impact on the level of miR-488 and miR-29c-3p expression, and there are significant differences between groups (*P* < 0.05), as detailed in Table 4. Based on the expression levels of GDF15 protein, the patients could be categorized as two groups: high expression (*n* = 108) and low expression (*n* = 92). In addition, the depth of invasion, TNM stage, and lymph node metastasis could affect the level of GDF15 expression in patients with colon cancer, and there were significant differences between the two groups (*P* < 0.05), as detailed in Table 5.

## 4. Discussion

In the early stage of colon cancer, there are often transient abdominal pain, diarrhea, constipation, increased stool frequency, and so on [20–22]. Because the symptoms are not very typical, most patients miss the best time for treatment, and they are already in the middle and late stage, affecting the effect of treatment [19, 23]. In order to improve the diagnostic accuracy in the early stage and development of colon cancer, it is necessary to explore the relevant factors in order to determine the treatment plan.

MicroRNA is a kind of short-stranded noncoding RNA, in clinic, which has a certain effect in regulating the progression of disease [24, 25]. According to related studies, it has been found that overexpression of miR-488 can significantly improve the sensitivity of cancer cells to bladder cancer drugs, and then promote cancer cell apoptosis [26, 27]. In this study, the expression level of miR-488 in colon cancer tissues was significantly lower than that in adjacent tissues, suggesting that the abnormal expression of miR-488 can reflect the occurrence of colon cancer to some extent. In this study, the degree of differentiation, depth of invasion, TNM stage, lymph node metastasis, and other factors are closely related to the abnormal expression of miR-488, indicating that the low expression of this index reflects the development of colon cancer and poor prognosis to some extent. miR-29c-3p, also known as Dead Bone tablet, is one of the autophagy proteins, which can participate in the process of autophagy and apoptosis of tumor cells [28, 29]. According to related studies, compared with normal gastric mucosa, the positive rate of miR-29c-3p in gastric cancer tissue is higher than that in normal gastric mucosa [30, 31]. It is analyzed that the occurrence of this situation is closely related to tumor involvement in autophagy. In this study, comparing the miR-29c-3p expression level and high expression rate in colon cancer tissue with that in adjacent tissues, we can find that the higher degree of differentiation, depth of invasion, TNM stage, lymph node metastasis, and other factors have influence on the index changes, suggesting that the abnormal index is related to its participation in the occurrence and development of colon cancer by participating in the process of autophagy, which can more accurately reflect the progression of colon cancer. According to related studies, compared with normal hepatocytes, the expression of this index in hepatocellular carcinoma cells is higher, indicating that the expression of GDF15 is closely related to the invasion and metastasis of dry-cleaning cells [32, 33]. Moreover, the increase of GDF15 protein in human prostate tissue can promote the growth of prostate tumors and cancer cells to a certain extent [34, 35]. In this study, the expression level of GDF15 mRNA and the high expression rate of GDF15 protein were higher in colon cancer, suggesting that GDF15 may be involved in the progression of colon cancer.

The article "Effect of miR-488 on Colon Cancer Biology and Clinical Applications" was retracted in 2023. Reasons: signs of a paper mill; compromised peer review; unreliable results or conclusions.

To sum up, compared with the adjacent tissues, the expression of miR-488 in colon cancer tissues was downregulated, while the high expression rates of miR-29c-3p and GDF15 mRNA were upregulated, and the three indexes were closely related to the depth of invasion, TNM stage, and lymph node metastasis. In this study, we can draw a preliminary conclusion that miR-129-5 and miR-29c-3p may affect the progression and prognosis of patients with colon cancer by regulating the expression of GDF15, but the specific mechanism still needs to be analyzed and studied in detail.

## Figures and Tables

**Table 1:** Relative expressions of miR-488, miR-29c-3p, and GDF15 mRNA in different colonic tissues ($\bar{x}\pm s$).

Tissue classification	*n*	miR-488 (U6)	miR-29c-3p (*β*-actin)	GDF15 mRNA (*β*-actin)

Colon cancer tissue	200	0.70 ± 0.24	2.79 ± 0.95	4.36 ± 1.42
Paracancerous tissue	200	1.05 ± 0.33	1.02 ± 0.28	1.01 ± 0.32
*t*	—	12.130	25.274	32.547
*P* value	—	<0.001	<0.001	<0.001

**Table 2:** Expression of miR-29c-3p and GDF15 in different colonic tissues (*n* (%)).

Tissue classification	*n*	miR-29c-3p			GDF15 protein		
		High expression	Low expression	High expression rate	High expression	Low expression	High expression rate

Colon cancer tissue	200	121	79	60.50	137	63	68.50
Paracancerous tissue	200	78	122	39.00	57	143	28.50
*χ* ^2^	—	—	—	18.490	—	—	64.058
*P* value	—	—	—	<0.001	—	—	<0.001

**Table 3:** Relationship between expression of miR-488 and clinicopathological features of colon cancer (*n* (%)).

Clinical pathological characteristics	*n*	miR-488		*χ* ^2^	*P* value
		High expression (*n* = 118)	Low expression (*n* = 82)		

Gender					
Male	106	56	50	3.549	0.060
Female	94	62	32		
Age					
<54	102	56	46	1.445	0.229
≥54	98	62	36		
Tumor location					
Left colon	101	63	38	0.961	0.327
Right colon	99	55	44		
Tumor diameter					
<5 cm	107	69	38	2.863	0.091
≥5 cm	93	49	44		
Degree of differentiation					
Highly-middle differentiation	112	63	49	0.796	0.372
Low differentiation	88	55	33		
Infiltration depth					
T1-T2	114	78	36	9.727	0.002
T3-T4	86	40	46		
TNM stage					
I-II	105	69	36	4.120	0.042
III	95	49	46		
Lymph node metastasis					
No	113	79	34	12.786	<0.001
Yes	87	39	48		

**Table 4:** Relationship between expression of miR-29c-3p and clinicopathological features of colon cancer.

Clinical pathological characteristics	*n*	miR-29c-3p		*χ* ^2^	*P* value
		High expression (*n* = 113)	Low expression (*n* = 87)		

Gender					
Male	106	56	50	1.236	0.266
Female	94	57	37		
Age					
<54	102	55	47	0.563	0.453
≥54	98	58	40		
Tumor location					
Left colon	101	62	39	1.982	0.159
Right colon	99	51	48		
Tumor diameter					
<5 cm	107	59	48	0.173	0.667
≥5 cm	93	54	39		
Degree of differentiation					
Highly-middle differentiation	112	57	55	0.203	0.379
Low differentiation	88	66	22		
Infiltration depth					
T1-T2	114	75	39	9.309	0.002
T3-T4	86	38	48		
TNM stage					
I-II	105	70	35	9.296	0.002
III	95	43	52		
Lymph node metastasis					
No	113	76	37	12.229	<0.001
Yes	87	37	50		

**Table 5:** Relationship between GDF15 protein and clinicopathologic features of colon cancer.

Clinical pathological characteristics	*n*	GDF15 protein		*χ* ^2^	*P* value
		High expression (*n* = 108)	Low expression (*n* = 92)		

Gender					
Male	106	60	46	0.616	0.433
Female	94	48	46		
Age					
<54	102	52	50	0.764	0.382
≥54	98	56	42		
Tumor location					
Left colon	101	59	42	1.602	0.206
Right colon	99	49	50		
Tumor diameter					
<5 cm	107	53	54	1.849	0.174
≥5 cm	93	55	38		
Degree of differentiation					
Highly-middle differentiation	112	58	54	0.502	0.478
Low differentiation	88	50	38		
Infiltration depth					
T1-T2	114	81	33	31.036	<0.001
T3-T4	86	27	59		
TNM stage					
I-II	105	77	28	33.263	<0.001
III	95	31	64		
Lymph node metastasis					
No	113	69	44	5.215	0.022
Yes	87	39	48		

The article "Effect of miR-488 on Colon Cancer Biology and Clinical Applications" was retracted in 2023. Reasons: signs of a paper mill; compromised peer review; unreliable results or conclusions.

## Data Availability

The analyzed data sets generated during the study are available from the corresponding author on reasonable request.
